# Obesity as a Consequence of Gut Bacteria and Diet Interactions

**DOI:** 10.1155/2014/651895

**Published:** 2014-03-06

**Authors:** Katerina Kotzampassi, Evangelos J. Giamarellos-Bourboulis, George Stavrou

**Affiliations:** ^1^Department of Surgery, Medical School, Aristotle University of Thessaloniki, Thessaloniki 54006, Greece; ^2^Fourth Department of Internal Medicine, University of Athens Medical School, Athens 12462, Greece

## Abstract

Obesity is a major public health concern, caused by a combination of increased consumption of energy-dense foods and reduced physical activity, with contributions from host genetics, environment, and adipose tissue inflammation. In recent years, the gut microbiome has also been found to be implicated and augmented research in mice and humans have attributed to it both the manifestation and/or exacerbation of this major epidemic and vice versa. At the experimental level, analysis of fecal samples revealed a potential link between obesity and alterations in the gut flora (drop in Bacteroidetes and increase in Firmicutes), the specific gut microbiome being associated with the obese phenotype. Conventionally raised mice were found to have over 40% more total body fat compared with those raised under germ-free conditions, while conventionalization of germ-free mice resulted in a significant increase in total body fat. Similarly, the sparse data in humans supports the fact that fat storage is favoured by the presence of the gut microbiota, through a multifaceted mechanism. Efforts to identify new therapeutic strategies to modulate gut microbiota would be of high priority for public health, and to date, probiotics and/or prebiotics seem to be the most effective tools.

## 1. Introduction

Obesity is a major public health concern, threatening both the industrialized and the developing countries, largely in parallel to the adoption of a “modern”/Western-type lifestyle. It results from a long-term disbalance between energy intake and expenditure, that is, increased consumption of more energy-dense, nutrient-poor foods containing high levels of sugar and saturated fats in combination with reduced physical activity [1]. However, the mechanisms underlying obesity seem to be far from the long-held belief in caloric intake and lifestyle factors. It is becoming evident that obesity and its causes are significantly more complex than previously thought, with contributions from host genetics, environment, diet and lifestyle, and systemic and adipose tissue inflammation [2].

Obesity is now characterized by a cluster of important chronic metabolic disorders, including insulin resistance, type 2 diabetes, fatty liver disease, atherosclerosis, hypertension, and hypercholesterolemia, and by a low grade of systemic inflammation [3], being the cause of exacerbation of all the above and leading to increased morbidity and mortality. Moreover, obesity is detrimental to the quality of life as a whole and implies high health costs as a consequence of its associated morbidities.

In recent years, augmented research worldwide has focused on the implication of intestinal microbiota in both the manifestation and exacerbation of this major epidemic and vice versa.

## 2. Obesity and Microbiota

Recent studies have suggested microbiota to be an environmental factor involved in the control of body weight and energy homeostasis. Experimental models using transgenic, knockout, and gnotobiotic animals, as well as human studies, provide evidence of a crucial role for intestinal microbiota in energy harvest and consequently obesity. More precisely, they show a potential link between obesity and alterations in the gut flora [4, 5], the specific gut microbiome being associated with the obese phenotype [5–10].

It is now well documented that the human gut microbiota (a total of up to 100 trillion cells), mostly Gram-positive and anaerobic [11], are unique to each individual, highly variable between persons, and remarkably stable after the first year of life [12, 13]. Despite this individual uniqueness and the high diversity in humans, there is only a small number of microbial phyla that are numerically dominant [14–16]: Firmicutes and Bacteroidetes accounting for more than 90% [17–19].

New research reveals that obese animal and human subjects have alterations in the composition of the gut microbiota compared to their leaner counterparts [20]; a greater representation of Firmicutes and fewer Bacteroidetes, as well as reduced bacterial diversity as a total [4, 5, 21, 22], the altered representation of bacterial genes being considered the cause affecting metabolic pathways [21].

In a challenge to identify more specific changes in the gut microbiota that may account for these metabolic effects, Ley et al. [5] studied genetically obese, leptin receptor-deficient (ob/ob) mice and found in the cecum biota a 50% reduction in the abundance of Bacteroidetes and a proportional increase in Firmicutes in relation to lean mice. Another researcher also found a higher proportion of Archaea microbes within the stools received from the cecum in genetically obese mice in comparison with their lean littermates [23], while diet-induced obesity in mice has also been associated with an increased proportion of* Eubacterium dolichum*, belonging to the Firmicutes division [24].

Waldram et al. [22] studied a rat obesity model, characterizing gut microbiotas in parallel with metabolites. Their results broadly support patterns of greater Firmicutes/Bacteroidetes ratios, as observed in other animal studies. Furthermore, specific bacteria were found associated with the obese phenotype (*Halomonas* and* Sphingomonas*), as were lower total bacteria counts and lower bifidobacterial counts. On the other hand, conventionally raised mice had over 40% more total body fat compared with those raised under germ-free conditions, while conventionalization of germ-free mice via colonization with cecum-derived distal microbial community resulted in a significant increase in total body fat [4].

The first study describing qualitative changes of the gut microbiota in obese human individuals over lean controls was published a few years ago [5, 9]. It analyzes the fecal gut microbiota over the course of 1 year in obese individuals participating in a weight loss programme, randomly allocated to either a fat-restricted or carbohydrate-restricted low-calorie diet. The Bacteroidetes and Firmicutes phyla were found to be the dominated microbiota, while bacterial flora showed remarkable intraindividual stability over time. At zero time-point, obese subjects had significantly fewer Bacteroidetes and more Firmicutes than lean control subjects. After weight loss, the relative proportion of Bacteroidetes increased, while Firmicutes decreased, a finding which is well correlated to the percentage of weight loss. Bacteroidetes constituted approximately 3% of the gut bacteria before diet therapy and approximately 15% after successful weight loss.

In another study on obese humans submitted to a dietary intervention of reduced carbohydrate intake and increased protein intake, Duncan et al. [25] found reductions in populations of* Bifidobacterium*,* Roseburia* spp., and* Eubacterium rectale*  subgroups of clostridial cluster XIVa. Further support derived from other weight loss studies show marked and sustained changes in the microbial composition of the gut after weight loss induced by diet restriction [26, 27]. In line with these findings were those obtained from individuals subjected to weight loss surgery [28–31]. Zhang et al. [28] showed that Gamma-Proteobacteria and Verrucomicrobia were enriched after gastric bypass compared with that presenting in the stools of lean and obese controls, while Firmicutes was significantly decreased. In addition, the stomach chambers formed in Roux-en-Y gastric bypass (RYGB) surgery are colonized by bacteria to a greater extent than in the normal stomach [31].

The hypothesis of a more specific modulation of gut microbiota in obesity, far from that obtained at the phylum levels, is supported by several studies.* Bifidobacterium* spp. numbers were found higher in children who exhibited a normal weight from birth till the age of 7 years in relation to children who became overweight [32], and is it now well known that* Bifidobacterium* spp. presence is often associated with beneficial health effects [33–35]. More importantly, the authors [32] observed that the* Staphylococcus aureus* levels were lower in children who maintained a normal weight than in children who became overweight several years later and thus proposed that the protection from obesity seen with bifidobacteria may, in part, be due to its anti-inflammatory effects, whereas* S. aureus* may trigger low-grade inflammation [36], leading to the overweight status [37, 38]. Furthermore, comparable results have been found between the faecal microbiota of obese and lean twins: while a core gut microbiome exists in both subjects, obese individuals exhibit reduced diversity and an altered representation of metabolic pathways in their microbiota [39], in addition to the lower proportion of Bacteroidetes and the higher proportion of Actinobacteria associated with obesity [21].

## 3. What Is the Role of Food Intake?

One of the key and central questions is that whether and how diet might affect the composition of the gut microbiome. In a very recent paper Emeritus Professor Bengmark [1], well known for his extensive studies on probiotics, summarizes the role of food as follows: “The great majority of ingredients in the industrially produced foods consumed in the West are absorbed in the upper part of small intestine and thus of limited benefit to the microbiota. Lack of proper nutrition for microbiota is a major factor under-pinning dysfunctional microbiota, dysbiosis, chronically elevated inflammation, and the production and leakage of endotoxins through the various tissue barriers. Furthermore, the over-consumption of insulinogenic foods and proteotoxins, such as advanced glycation and lipoxidation molecules, gluten and zein, and a reduced intake of fruit and vegetables, are key factors behind the commonly observed elevated inflammation and the endemic of obesity and chronic diseases, factors which are also likely to be detrimental to microbiota.” The fact that industrialized foods are absorbed in the upper part of the small intestine, in relation to the knowledge that lactobacilli are predominantly present in the ileum and bifidobacteria in the colon [40] would be a simplified explanation for lactobacilli overgrowth and bifidobacteria suppression in obese individuals.

On the other hand, the finding of increase in fat mass upon high-fat diet feeding in conventionalized versus germ-free animals supports the fact that the fat storage is favoured by the presence of gut microbiota [4, 7] and that carbohydrates in the diet may modulate the development of obesity upon colonization of the gut as well [41].

At experimental level, Hildebrandt et al. [42] focused on how a high-fat diet might affect the composition of the murine gut microbiome, even independently of obesity. When switching mice to a high-fat diet, they found profound changes in the gut microbiome, including a decrease in Bacteroidetes and an increase in Firmicutes and Proteobacteria. However, the main strength of their study is that they clearly show the observed changes to be independent of obesity.

In an effort to ascertain to what extent gut microbiota is an important regulator of nutrient absorption in humans, Jumpertz et al. [40] investigated the changes in the feces of 12 lean and 9 obese individuals during diets that varied in caloric content (2400 compared with 3400 kcal/d). They showed that an altered nutrient load induced rapid changes in the bacterial composition of the human gut microbiota. Moreover, these changes in the gut microbiota were directly associated with stool energy loss in lean individuals, such that a 20% increase in Firmicutes and a corresponding decrease in Bacteroidetes were associated with an increased energy harvest of about 150 kcal. They also showed that a high degree of overfeeding in lean subjects was associated with a greater fractional decrease in stool energy loss, which indicated that the degree of overnutrition relative to individual weight-maintaining energy needs may have played a role in the determination of the efficiency of nutrient absorption and may potentially explain the observation of clearer associations in lean compared with obese subjects. Thus, they suggest that the gut microbiota senses alterations in nutrient availability and subsequently modulates nutrient absorption, the difference in microbiota reflecting differences in calorie absorption. Moreover, previous studies on healthy subjects showed that about 5% of ingested calories were lost in stools [43], with those consuming high-fiber diets exhibiting a higher fecal energy loss than those consuming a low-fiber diet, although equivalent in energy content [44, 45].

The change of the composition of the upper intestine in obesity for aerobic bacteria was also confirmed in a survey of 320 patients subject to upper GI tract endoscopy. Fluid was aspirated from the lumen of the third part of the duodenum and it was quantitatively cultured. The isolation of colonic type bacteria at counts greater than 10^3^ cfu/mL was considered diagnostic of the syndrome of intestinal bacterial overgrowth (SIBO). SIBO was present among 62 patients. When patients with SIBO were compared with the 258 non-SIBO patients regarding their baseline demographic characteristics, it was found that the BMI of SIBO patients was significantly greater than that of non-SIBO patients (mean 28.2 kg/m^2^ versus 25.1 kg/m^2^). As expected, the prevalence of type 2 diabetes mellitus was far greater among SIBO patients than among non-SIBO patients (25.5% versus 18.2%) [46].

## 4. Mechanisms Involved in Fat Storage

From all the above described findings, it appears clear that gut microbiota is an important environmental factor that affects energy harvest from the diet and energy storage in the host [4], through a multiple-faceted mechanism regulating the host's metabolism.

First of all, gut microbiota seems to promote fat storage by means of linking circulating triglycerides with suppression of the intestinal expression of an inhibitor of lipoprotein lipase (LPL) [4], the so-called fasting-induced adipose factor (Fiaf). This is member of the angiopoietin-like family of proteins, expressed in differentiated gut epithelial cells, as well as in the liver and the adipose tissue [47], which is considered to be a mediator of microbial regulation of energy storage [4]. Further research on germ-free and conventionalized, normal and Fiaf knockout mice has established its essential role for the microbiota-induced deposition of triglycerides in adipocytes [4, 10] by means of LPS activity. Gut microbiota-induced suppression of Fiaf leads to a higher LPL activity and as a consequence an increased cellular uptake of fatty acids and adipocyte triglyceride accumulation, that is, greater fat storage [4]. It is likely that changes in gut microbial environment prompted by Western diets may function as an “environmental” factor that affects predisposition toward energy storage and obesity [4]. On the other hand, it would appear logical to try modulating gut flora towards increasing Fiaf expression and or activity, an action that would promote leanness.

A second pathway that influences host energy storage is related to energy extraction from undigested food components. Nutrients which escape the digestion, due to host's limited capability of glycoside hydrolases to digest complex dietary plant polysaccharides, are fermented by gut microbes into monosaccharides and short-chain fatty acids (SCFAs), such as acetate, propionate, and butyrate [11, 48], representing an important energy source for the body. Normal colonic epithelia derive 60–70% of their energy supply from SCFAs, particularly butyrate [49, 50], while propionate is largely taken up by the liver for gluconeogenesis, liponeogenesis, and protein synthesis [51, 52].

Changes in the relative abundance of the two dominant bacterial phyla, the Bacteroidetes and Firmicutes, found in obese mice and humans, are associated with differences in capacity for energy harvest [4, 5]. The increase of microbiota phyla such as “obese gut microbiome” with greater energy extraction efficiency resulted in less energy left over in feces and thus greater levels of short-chain fatty acids (SCFAs) in the cecum.

Schwiertz et al. [53] found considerable differences in the stool SCFAs' concentrations between lean and obese individuals; the mean total SCFA concentration in fecal samples of obese volunteers was more than 20% higher in total than in lean volunteers (*P* = 0.024); the highest increase is seen for propionate with 41% (*P* = 0.002), followed by butyrate (28%, *P* = 0.095). In addition, this resulted in changes in the proportions of individual to total SCFA, the propionate proportion was thus higher in overweight (18.7%, *P* = 0.019) and obese (18.3%, *P* = 0.028) than in lean subjects (15.9%).

SCFAs may also act as signalling molecules, since propionate and acetate are known ligands for 2 G-protein-coupled receptors (GPCRs), namely, the Gpr41 and Gpr43 [54, 55]. Thus, manipulation of SCFA activation of GPCRs could, theoretically, serve as a therapeutic target, modulating efficiency of caloric extraction from a polysaccharide-rich diet.

In addition to the effect on energy harvest, the bacterial microbiota can directly, via afferent nerve terminals or indirectly, via signalling peptides, modulate gut motility, alter secretion of gut hormones, and modify both gut permeability and immune function. These alterations may additionally influence the host metabolism and proinflammatory state being present in obesity [56].

A 4-week high-fat diet in a mouse model appears to increase the proportion of circulating lipopolysaccharide- (LPS-) containing microbiota [38] and thus plasma LPS levels (metabolic endotoxemia) two to threefold. Thus, a high-fat diet is thought to modulate the composition of the gut bacteria [24, 57–59] (notably by reducing bifidobacteria), leading to increase in gut permeability which allows a higher LPS plasma levels. On the other hand, greater levels of bifidobacteria have been associated with reduced gut leakiness, allowing less LPS to translocate to the serum [60].

Cani et al. [4, 59] have recently shown that an increase of LPS levels, derived from colonic Gram-negative bacteria, such as the Bacteroidetes which, in association with and/or due to changes in intestinal microbiota composition (gram-negative/gram-positive ratio), seems to be a triggering factor in chronic systemic inflammation; an increased production of proinflammatory cytokines affects negatively glucose tolerance and thus leads to insulin resistance and increase in body weight. More precisely, it is well known that LPS binding to TLR4 receptor triggers a downstream signaling cascade that encodes proinflammatory molecules. Shi et al. [61] have shown that nutritional fatty acids, whose circulating levels are often increased in obesity, activate TLR4 signaling in adipocytes and macrophages in a similar way, the chronic inflammatory state being associated with insulin resistance.

Additionally, when mice received a high-fat diet plus antibiotics, they are found to have decreased levels of endotoxin and decreased markers of inflammation, as well as reduced weight gain and improved glucose tolerance [59], a finding implying that LPS may link inflammation with the microbiota. Thus, the manipulation of the gut microbiota may provide a novel therapeutic treatment for obesity [62–64].

Another pathway of potential interaction between host and the microbiota involves the adenosine monophosphate-activated protein kinase (AMPK), a key enzyme that controls cellular energy status through stimulation of fatty acids beta-oxidation [7, 10, 65]. The gut microbiotas were found to suppress AMPK-driven fatty acid oxidation in the liver and in skeletal muscle, while germ-free mice remain lean, despite high calorie intake, due to increased activity of AMPK levels both in the liver and skeletal muscle, which stimulate fatty acid and lead to decreased glycogen levels in the liver [7].

Finally, Stappenbeck et al. [66] suggested that gut microbiota conventionalization in mice results in a doubling of the density of capillaries in the villus epithelium of the small intestine, in an effort to promote intestinal monosaccharide absorption.

## 5. Future Perspectives

The ability to extract energy from every kind of food and to store it as adipose tissue would be a beneficial attribute for our ancestors who had variable access to food around the year. Nowadays, in our modern, developed world, where there is ready access to inexpensive, large-portion, readily available high-calorie foods, this “benefit” becomes a disadvantage, with overweight and obesity representing major risk factors for a plethora of severe metabolic disorders, including dyslipidemia, steatosis, hypertension, insulin resistance and type 2 diabetes, cardiovascular diseases, and inflammatory bowel diseases.

However, most obese individuals have been found unable to make voluntary, lifelong changes in diet and behaviour for weight management. Moreover, very recent laboratory and clinical research has documented that excessive fat accumulation is the consequence not only of positive energy balance and decreased physical activity affected by cultural and economic factors. Major progress has been made in identifying specific nutrition components that are both directly linked to the inflammatory state of the host and dramatically shift the assemblage of gut microbiota, whichever the order of priority [67].

As has already been analyzed, at the phyla level, Firmicute dominant, “obese” microbiomes were found to contain more genes associated with lipid and carbohydrate metabolism and the breakdown of otherwise indigestible polysaccharides than Bacteroidetes dominant, the “lean” microbiomes did [37]. Therefore, efforts to identify new therapeutic strategies allowing noncognitive reduction of energy intake, energy absorption, and storage would be of high priority for public health, the most prominent target being the restoration of the gut microbiota to a healthy state. What are the next logical steps? We should search for certain dietary or pharmacological interventions to manipulate specific gut microbial species [6, 24, 55, 68].

Among the tools to modulate gut microbiota, probiotics and/or prebiotics appear to be the most important, although actual proof is still limited. The Food and Agriculture Organization of the United Nations and the World Health Organization (FAO/WHO) define probiotics as “live microorganisms that, when ingested in adequate quantities, exert a health benefit to the host,” by stimulating the growth of other microorganisms, modulating mucosal and systemic immunity, and improving the nutritional and microbial balance in the intestinal tract [69]. On the other hand, prebiotics are nondigestible food ingredients that beneficially affect the host by selectively stimulating the growth and/or activity of one or a limited number of the host's gut bacteria [70].

Various probiotic strains have already been evaluated as therapeutic in animal models of obesity, such as* Bifidobacterium* spp. [71, 72],* Lactobacillus paracasei* [73], and* Lactobacillus gasseri* BNR17 [74]. In humans, although actual proof is still limited, the few human trials are encouraging and seem to be very promising with regard to the efficacy of pre- and/or probiotics as antiobesity agents [75–77]. The early modulation of gut microbiota with the probiotics* Lactobacillus rhamnosus* GG and* Bifidobacterium lactis* Bb12 was found to reduce the body mass index in young children, by restraining excessive weight gain during the first 10 years of life [78]. Sixty-two obese volunteers were randomized into* Lactobacillus gasseri* BNR17 or placebo for a 12-week period, at the end of which a slight reduction in body weight and a decrease of waist and hip circumferences were noted in the BNR17 group, the nonsignificant difference being attributed to the short trial period [79]. The effect of the probiotic* Lactobacillus gasseri* SBT2055 (LG2055) was tested in 87 obese subjects, in a randomized, placebo controlled intervention which lasted 12 weeks. A significant decrease in body weight and body mass index as well as in visceral and subcutaneous fat was found, which may be linked to decreased fat absorption in relation to the control group [80].

Giving inulin-type fructooligosaccharides (FOS) as a supplement seems to stimulate the growth of* Bifidobacterium* spp. and, in some cases,* Lactobacillus* spp., which are also administrated as probiotics [81–83]. Similarly, wheat arabinoxylan was found related to consistent increases in Bacteroidetes, bifidobacteria, and* Roseburia* [84]. It is of interest to mention that the amount of Bifidobacteria found at baseline (i.e., before intervention) seems to be strongly associated with the increase achieved after treatment, indicating that preexistent gut microbiota composition enhances or possibly determines the response to the intervention [56]. Oligofructose supplementation (21 g daily) versus maltodextrin as placebo for a 12-week period in 48 healthy obese adults was found to promote weight loss and improve glucose regulation, through a modulation of satiety hormone concentrations leading to the reduction in energy intake [85].

The consumption of a symbiotic food, for one month, containing fructooligosaccharides and the probiotic strains* Lactobacillus helveticus* Bar13 and* Bifidobacterium longum* Bar33, was tested in 20 healthy subjects. The intake of the synbiotic food demonstrated no modification on the overall structure of the gut microbiome but resulted in a shift of the fecal metabolic profiles, that is, a significant increase of SCFA, ketones, carbon disulfide, and methyl acetate, suggesting potential health promoting effects [86].

In a recent randomized controlled study on 65 mechanically ventilated trauma patients it was shown that the synbiotic formula Synbiotic 2000FORTE (Medipharm, Kågeröd, Sweden), being a preparation of* Pediococcus pentosaceus* 5-33:3,* Leuconostoc mesenteroides* 32-77:1,* Lactobacillus paracasei* ssp. 19 and* Lactobacillus plantarum* 2362, plus inulin, oat bran, pectin, and resistant starch as prebiotics, administered orally for 15 days versus maltodextrin as placebo, altered the composition of gut flora in favour of anaerobes [87]. In another randomized, double-blind trial, a beverage fermented with* L. acidophilus* and* Propionibacterium freudenreichii* was given to 43 healthy female subjects in order to study the satiety-inducing effects. Subjects exhibited a nonsignificant decreasing trend in ad libitum food consumption, but felt significantly fuller (*P* = 0.02), were less hungry (*P* = 0.004) and had less desire to eat (*P* = 0.006) after consumption of the fermented dairy beverage. The appetite-decreasing effects were ascribed to the production of propionate by* P. freudenreichii* [88]. Similarly, a decrease in appetite and an increase in satiety, leading to a decrease in total energy intake, as well as a decrease in hepatic de novo lipogenesis, have been demonstrated in human volunteers fed with inulin-type prebiotics (16 g daily) versus maltodextrin as a control [89].

Finally, the success in faecal transplantation for* C. difficile* diarrhoea treatment [90, 91] gives promising results for a new era involving transplantation of stools from lean subjects to achieve weight loss.

In summary, ongoing research on human gut microbiota seems, in the short term, to allow the positive manipulation of the interior milieu of a human being by means of either the appropriate microbiome exhibiting antiobesity effects and/or the right substrate (prebiotic) to promote its growth.

## References

[1] Bengmark S (2013). Gut microbiota, immune development and function. *Pharmacological Research*.

[2] Maury E, Brichard SM (2010). Adipokine dysregulation, adipose tissue inflammation and metabolic syndrome. *Molecular and Cellular Endocrinology*.

[3] Pataky Z, Bobbíoni-Harsch E, Hadengue A, Carpentier A, Golay A (2009). Gut microbiota, responsible for our body weight?. *Revue Medicale Suisse*.

[4] Bäckhed F, Ding H, Wang T (2004). The gut microbiota as an environmental factor that regulates fat storage. *Proceedings of the National Academy of Sciences of the United States of America*.

[5] Ley RE, Bäckhed F, Turnbaugh P, Lozupone CA, Knight RD, Gordon JI (2005). Obesity alters gut microbial ecology. *Proceedings of the National Academy of Sciences of the United States of America*.

[6] Turnbaugh PJ, Ley RE, Mahowald MA, Magrini V, Mardis ER, Gordon JI (2006). An obesity-associated gut microbiome with increased capacity for energy harvest. *Nature*.

[7] Bäckhed F, Manchester JK, Semenkovich CF, Gordon JI (2007). Mechanisms underlying the resistance to diet-induced obesity in germ-free mice. *Proceedings of the National Academy of Sciences of the United States of America*.

[8] Delzenne NM, Cani PD (2011). Interaction between obesity and the gut microbiota: relevance in nutrition. *Annual Review of Nutrition*.

[9] Ley RE, Turnbaugh PJ, Klein S, Gordon JI (2006). Microbial ecology: human gut microbes associated with obesity. *Nature*.

[10] Tennyson CA, Friedman G (2008). Microecology, obesity, and probiotics. *Current Opinion in Endocrinology, Diabetes and Obesity*.

[11] Bäckhed F, Ley RE, Sonnenburg JL, Peterson DA, Gordon JI (2005). Host-bacterial mutualism in the human intestine. *Science*.

[12] Costello EK, Lauber CL, Hamady M, Fierer N, Gordon JI, Knight R (2009). Bacterial community variation in human body habitats across space and time. *Science*.

[13] Reinhardt C, Reigstad CS, Bäckhed F (2009). Intestinal microbiota during infancy and its implications for obesity. *Journal of Pediatric Gastroenterology and Nutrition*.

[14] Zoetendal EG, Vaughan EE, De Vos WM (2006). A microbial world within us. *Molecular Microbiology*.

[15] Zoetendal EG, Rajilić-Stojanović M, de Vos WM (2008). High-throughput diversity and functionality analysis of the gastrointestinal tract microbiota. *Gut*.

[16] Ley RE, Knight R, Gordon JI (2007). The human microbiome: eliminating the biomedical/environmental dichotomy in microbial ecology. *Environmental Microbiology*.

[17] Hugenholtz P, Goebel BM, Pace NR (1998). Impact of culture-independent studies on the emerging phylogenetic view of bacterial diversity. *Journal of Bacteriology*.

[18] Eckburg PB, Bik EM, Bernstein CN (2005). Microbiology: diversity of the human intestinal microbial flora. *Science*.

[19] Ley RE, Hamady M, Lozupone C (2008). Evolution of mammals and their gut microbes. *Science*.

[20] Bercik P, Collins SM, Verdu EF (2012). Microbes and the gut-brain axis. *Neurogastroenterology and Motility*.

[21] Turnbaugh PJ, Hamady M, Yatsunenko T (2009). A core gut microbiome in obese and lean twins. *Nature*.

[22] Waldram A, Holmes E, Wang Y (2009). Top-down systems biology modeling of host metabotype-microbiome associations in obese rodents. *Journal of Proteome Research*.

[23] Samuel BS, Hansen EE, Manchester JK (2007). Genomic and metabolic adaptations of Methanobrevibacter smithii to the human gut. *Proceedings of the National Academy of Sciences of the United States of America*.

[24] Turnbaugh PJ, Bäckhed F, Fulton L, Gordon JI (2008). Diet induced obesity is linked to marked but reversible alterations in the mouse distal gut microbiome. *Cell Host and Microbe*.

[25] Duncan SH, Belenguer A, Holtrop G, Johnstone AM, Flint HJ, Lobley GE (2007). Reduced dietary intake of carbohydrates by obese subjects results in decreased concentrations of butyrate and butyrate-producing bacteria in feces. *Applied and Environmental Microbiology*.

[26] Santacruz A, Marcos A, Wärnberg J (2009). Interplay between weight loss and gut microbiota composition in overweight adolescents. *Obesity*.

[27] Nadal I, Santacruz A, Marcos A (2009). Shifts in clostridia, bacteroides and immunoglobulin-coating fecal bacteria associated with weight loss in obese adolescents. *International Journal of Obesity*.

[28] Zhang H, DiBaise JK, Zuccolo A (2009). Human gut microbiota in obesity and after gastric bypass. *Proceedings of the National Academy of Sciences of the United States of America*.

[29] Furet JP, Kong LC, Tap J (2010). Differential adaptation of human gut microbiota to bariatric surgery-induced weight loss: links with metabolic and low-grade inflammation markers. *Diabetes*.

[30] Li JV, Ashrafian H, Bueter M (2011). Metabolic surgery profoundly influences gut microbial—host metabolic cross-talk. *Gut*.

[31] Ishida RK, Faintuch J, Paula AMR (2007). Microbial flora of the stomach after gastric bypass for morbid obesity. *Obesity Surgery*.

[32] Kalliomäki M, Collado MC, Salminen S, Isolauri E (2008). Early differences in fecal microbiota composition in children may predict overweight. *The American Journal of Clinical Nutrition*.

[33] Boesten RJ, Schuren FHJ, de Vos WM (2009). A bifidobacterium mixed-species microarray for high resolution discrimination between intestinal bifidobacteria. *Journal of Microbiological Methods*.

[34] Turroni F, Marchesi JR, Foroni E (2009). Microbiomic analysis of the bifidobacterial population in the human distal gut. *ISME Journal*.

[35] Boesten RJ, de Vos WM (2008). Interactomics in the human intestine: lactobacilli and bifidobacteria make a difference. *Journal of clinical gastroenterology*.

[36] Lundell AC, Adlerberth I, Lindberg E (2007). Increased levels of circulating soluble CD14 but not CD83 in infants are associated with early intestinal colonization with Staphylococcus aureus. *Clinical and Experimental Allergy*.

[37] Kaplan JL, Walker WA (2012). Early gut colonization and subsequent obesity risk. *Current Opinion in Clinical Nutrition and Metabolic Care*.

[38] Cani PD, Amar J, Iglesias MA (2007). Metabolic endotoxemia initiates obesity and insulin resistance. *Diabetes*.

[39] Tilg H (2010). Obesity, metabolic syndrome and microbiota: multiple interactions. *Journal of Clinical Gastroenterology*.

[40] Jumpertz R, Le DS, Turnbaugh PJ (2011). Energy-balance studies reveal associations between gut microbes, caloric load, and nutrient absorption in humans. *The American Journal of Clinical Nutrition*.

[41] Fleissner CK, Huebel N, Abd El-Bary MM, Loh G, Klaus S, Blaut M (2010). Absence of intestinal microbiota does not protect mice from diet-induced obesity. *British Journal of Nutrition*.

[42] Hildebrandt MA, Hoffmann C, Sherrill-Mix SA (2009). High fat diet determines the composition of the murine gut microbiome independently of obesity. *Gastroenterology*.

[43] Beyer PL, Flynn MA (1978). Effects of high- and low-fiber diets on human feces. *Journal of the American Dietetic Association*.

[44] Wisker E, Maltz A, Feldheim W (1988). Metabolizable energy of diets low or high in dietary fiber from cereals when eaten by humans. *Journal of Nutrition*.

[45] Cliff Yoon J, Chickering TW, Rosen ED (2000). Peroxisome proliferator-activated receptor *γ* target gene encoding a novel angiopoietin-related protein associated with adipose differentiation. *Molecular and Cellular Biology*.

[46] Pyleris E, Giamarellos-Bourboulis EJ, Tzivras D, Koussoulas V, Barbatzas C, Pimentel M (2012). The prevalence of overgrowth by aerobic bacteria in the small intestine by small bowel culture: relationship with irritable bowel syndrome. *Digestive Diseases and Sciences*.

[47] Flint HJ, Bayer EA, Rincon MT, Lamed R, White BA (2008). Polysaccharide utilization by gut bacteria: potential for new insights from genomic analysis. *Nature Reviews Microbiology*.

[48] Mountzouris KC, Kotzampassi K, Tsirtsikos P, Kapoutzis K, Fegeros K (2009). Effects of Lactobacillus acidophilus on gut microflora metabolic biomarkers in fed and fasted rats. *Clinical Nutrition*.

[49] Scarpellini E, Campanale M, Leone D (2010). Gut microbiota and obesity. *Internal and Emergency Medicine*.

[50] Scheppach W (1994). Effects of short chain fatty acids on gut morphology and function. *Gut*.

[51] Wolever TMS, Spadafora P, Eshuis H (1991). Interaction between colonic acetate and propionate in humans. *The American Journal of Clinical Nutrition*.

[52] Vernay M (1987). Origin and utilization of volatile fatty acids and lactate in the rabbit: influence of the faecal excretion pattern. *British Journal of Nutrition*.

[53] Schwiertz A, Taras D, Schäfer K (2010). Microbiota and SCFA in lean and overweight healthy subjects. *Obesity*.

[54] Brown AJ, Goldsworthy SM, Barnes AA (2003). The orphan G protein-coupled receptors GPR41 and GPR43 are activated by propionate and other short chain carboxylic acids. *Journal of Biological Chemistry*.

[55] le Poul E, Loison C, Struyf S (2003). Functional characterization of human receptors for short chain fatty acids and their role in polymorphonuclear cell activation. *Journal of Biological Chemistry*.

[56] Diamant M, Blaak EE, de Vos WM (2011). Do nutrient-gut-microbiota interactions play a role in human obesity, insulin resistance and type 2 diabetes?. *Obesity Reviews*.

[57] Cani PD, Delzenne NM (2007). Gut microflora as a target for energy and metabolic homeostasis. *Current Opinion in Clinical Nutrition and Metabolic Care*.

[58] Cani PD, Hoste S, Guiot Y, Delzenne NM (2007). Dietary non-digestible carbohydrates promote L-cell differentiation in the proximal colon of rats. *British Journal of Nutrition*.

[59] Cani PD, Bibiloni R, Knauf C (2008). Changes in gut microbiota control metabolic endotoxemia-induced inflammation in high-fat diet-induced obesity and diabetes in mice. *Diabetes*.

[60] Cani PD, Possemiers S, van de Wiele T (2009). Changes in gut microbiota control inflammation in obese mice through a mechanism involving GLP-2-driven improvement of gut permeability. *Gut*.

[61] Shi H, Kokoeva MV, Inouye K, Tzameli I, Yin H, Flier JS (2006). TLR4 links innate immunity and fatty acid-induced insulin resistance. *Journal of Clinical Investigation*.

[62] Jia W, Li H, Zhao L, Nicholson JK (2008). Gut microbiota: a potential new territory for drug targeting. *Nature Reviews Drug Discovery*.

[63] Hoffman FA (2008). Development of probiotics as biologic drugs. *Clinical Infectious Diseases*.

[64] Membrez M, Blancher F, Jaquet M (2008). Gut microbiota modulation with norfloxacin and ampicillin enhances glucose tolerance in mice. *The FASEB Journal*.

[65] Kahn BB, Alquier T, Carling D, Hardie DG (2005). AMP-activated protein kinase: ancient energy gauge provides clues to modern understanding of metabolism. *Cell Metabolism*.

[66] Stappenbeck TS, Hooper LV, Gordon JI (2002). Developmental regulation of intestinal angiogenesis by indigenous microbes via Paneth cells. *Proceedings of the National Academy of Sciences of the United States of America*.

[67] Huang EY, Leone VA, Devkota S, Wang Y, Brady MJ, Chang EB (2013). Composition of dietary fat source shapes gut microbiota architecture and alters host inflammatory mediators in mouse adipose tissue. *Journal of Parenteral and Enteral Nutrition*.

[68] Cani PD, Neyrinck AM, Fava F (2007). Selective increases of bifidobacteria in gut microflora improve high-fat-diet-induced diabetes in mice through a mechanism associated with endotoxaemia. *Diabetologia*.

[69] Kotzampassi K, Giamarellos-Bourboulis EJ (2012). Probiotics for infectious diseases: more drugs, less dietary supplementation. *International Journal of Antimicrobial Agents*.

[70] Gibson GR, Probert HM, van Loo J, Rastall RA, Roberfroid MB (2004). Dietary modulation of the human colonic microbiota: updating the concept of prebiotics. *Nutrition Research Reviews*.

[71] Kondo S, Xiao JZ, Satoh T (2010). Antiobesity effects of bifidobacterium breve Strain B-3 supplementation in a mouse model with high-fat diet-Induced obesity. *Bioscience, Biotechnology and Biochemistry*.

[72] An HM, Park SY, Lee DK (2011). Antiobesity and lipid-lowering effects of Bifidobacterium spp. in high fat diet-induced obese rats. *Lipids in Health and Disease*.

[73] Aronsson L, Huang Y, Parini P (2010). Decreased fat storage by Lactobacillus paracasei is associated with increased levels of angiopoietin-like 4 protein (ANGPTL4). *PLoS ONE*.

[74] Kang JH, Yun SI, Park HO (2010). Effects of Lactobacillus gasseri BNR17 on body weight and adipose tissue mass in diet-induced overweight rats. *Journal of Microbiology*.

[75] Arora T, Singh S, Sharma RK (2013). Probiotics: interaction with gut microbiome and antiobesity potential. *Nutrition*.

[76] Robles Alonso V, Guarner F (2013). Linking the gut microbiota to human health. *British Journal of Nutrition*.

[77] Delzenne NM, Cani PD (2010). Nutritional modulation of gut microbiota in the context of obesity and insulin resistance: potential interest of prebiotics. *International Dairy Journal*.

[78] Luoto R, Laitinen K, Nermes M, Isolauri E (2010). Impact of maternal probiotic-supplemented dietary counselling on pregnancy outcome and prenatal and postnatal growth: a double-blind, placebo-controlled study. *British Journal of Nutrition*.

[79] Jung SP, Lee KM, Kang JH (2013). Effect of Lactobacillus gasseri BNR17 on overweight and obese adults: a randomized, double-blind clinical trial. *Korean Journal Of Family Medicine*.

[80] Kadooka Y, Sato M, Imaizumi K (2010). Regulation of abdominal adiposity by probiotics (Lactobacillus gasseri SBT2055) in adults with obese tendencies in a randomized controlled trial. *European Journal of Clinical Nutrition*.

[81] Bouhnik Y, Raskine L, Simoneau G (2004). The capacity of nondigestible carbohydrates to stimulate fecal bifidobacteria in healthy humans: a double-blind, randomized, placebo-controlled, parallel-group, dose-response relation study. *The American Journal of Clinical Nutrition*.

[82] Kolida S, Meyer D, Gibson GR (2007). A double-blind placebo-controlled study to establish the bifidogenic dose of inulin in healthy humans. *European Journal of Clinical Nutrition*.

[83] Macfarlane S, Macfarlane GT, Cummings JH (2006). Review article: prebiotics in the gastrointestinal tract. *Alimentary Pharmacology and Therapeutics*.

[84] Neyrinck AM, Possemiers S, Druart C (2011). Prebiotic effects of wheat Arabinoxylan related to the increase in bifidobacteria, roseburia and bacteroides/prevotella in diet-induced obese mice. *PLoS ONE*.

[85] Parnell JA, Reimer RA (2009). Weight loss during oligofructose supplementation is associated with decreased ghrelin and increased peptide YY in overweight and obese adults. *The American Journal of Clinical Nutrition*.

[86] Vitali B, Ndagijimana M, Cruciani F (2010). Impact of a synbiotic food on the gut microbial ecology and metabolic profiles. *BMC Microbiology*.

[87] Koutelidakis IM, Bezirtzoglou E, Giamarellos-Bourboulis EJ, Grosomanidis V, Kotzampassi K (2010). Impact of synbiotics on the intestinal flora of critically ill patients with multiple injuries. *International Journal of Antimicrobial Agents*.

[88] Ruijschop RMAJ, Boelrijk AEM, te Giffel MC (2008). Satiety effects of a dairy beverage fermented with propionic acid bacteria. *International Dairy Journal*.

[89] Cani PD, Lecourt E, Dewulf EM (2009). Gut microbiota fermentation of prebiotics increases satietogenic and incretin gut peptide production with consequences for appetite sensation and glucose response after a meal. *The American Journal of Clinical Nutrition*.

[90] Landy J, Al-Hassi HO, McLaughlin SD (2011). Review article: faecal transplantation therapy for gastrointestinal disease. *Alimentary Pharmacology and Therapeutics*.

[91] Borody TJ, Campbell J (2012). Fecal microbiota transplantation: techniques, applications, and issues. *Gastroenterology Clinics of North America*.

